# Health Conditions and Their Impact among Adolescents and Young Adults with Down Syndrome

**DOI:** 10.1371/journal.pone.0096868

**Published:** 2014-05-12

**Authors:** Terri J. Pikora, Jenny Bourke, Katherine Bathgate, Kitty-Rose Foley, Nicholas Lennox, Helen Leonard

**Affiliations:** 1 Telethon Kids Institute, The University of Western Australia, Perth, Western Australia, Australia; 2 School of Public Health, Curtin University, Bentley, Western Australia, Australia; 3 Queeensland Centre for Intellectual and Developmental Disability, University of Queensland, South Brisbane, Queensland, Australia; Rikagaku Kenkyūsho Brain Science Institute, Japan

## Abstract

**Objective:**

To examine the prevalence of medical conditions and use of health services among young adults with Down syndrome and describe the impact of these conditions upon their lives.

**Methods:**

Using questionnaire data collected in 2011 from parents of young adults with Down syndrome we investigated the medical conditions experienced by their children in the previous 12 months. Univariate, linear and logistic regression analyses were performed.

**Results:**

We found that in addition to the conditions commonly experienced by children with Down syndrome, including eye and vision problems (affecting 73%), ear and hearing problems (affecting 45%), cardiac (affecting 25%) and respiratory problems (affecting 36%), conditions also found to be prevalent within our young adult cohort included musculoskeletal conditions (affecting 61%), body weight (affecting 57%), skin (affecting 56%) and mental health (affecting 32%) conditions and among young women menstrual conditions (affecting 58%). Few parents reported that these conditions had no impact, with common impacts related to restrictions in opportunities to participate in employment and community leisure activities for the young people, as well as safety concerns.

**Conclusion:**

There is the need to monitor, screen and provide appropriate strategies such as through the promotion of healthy lifestyles to prevent the development of comorbidities in young people with Down syndrome and, where present, to reduce their impact.

## Introduction

With a relatively stable birth prevalence of almost one per 1000 live births in Western Australia over the past 20 years,[1] Down syndrome is the most common known cause of intellectual disability in developed countries.[2] Health-related problems occurring in children with Down syndrome include congenital heart[3], [4], [5] and gastrointestinal defects,[3], [4], [5] infections,[6], [7] ear and hearing impairments,[6], [8] thyroid disease,[7] childhood leukaemia,[9], [10] and immune-related disorders.[11] Age-related disorders also begin earlier in Down syndrome than in the general population. Adults with Down syndrome are at increased risk for skin and hair changes, early-onset menopause, visual and hearing losses,[12] adult-onset seizure disorder,[13] thyroid dysfunction,[14] diabetes,[15] obesity,[16] and musculoskeletal problems.[17] As life expectancy for individuals with Down syndrome has increased in infancy, childhood[18] and adulthood[19], [20] so has the incidence of dementia although development of Alzheimer's dementia is frequent but not inevitable.[21]. While research has investigated medical conditions among infants and children[4], [6], [22], [23], [24], [25] and older adults,[7], [26] medical issues among adolescents and young people with Down syndrome, who are at an important transition point in their lives, tend to have been neglected.

The aims of this paper were: to examine the prevalence of medical conditions and health service use among adolescents and young adults with Down syndrome; to describe the impact of these conditions upon the young person's daily life; and to explore the relationship between the presence of medical conditions and level of functioning in daily life.

## Methods

As part of an Australian-wide study of young adults with intellectual disability transitioning from school, young adults with Down syndrome were identified through the Western Australian (WA) Down Syndrome population database which has been following children with Down syndrome in Western Australia since 1997.[22], [23] In 2011 questionnaires were distributed to 223 families whose children were now young adults aged between 15 and 30 years. Approval for the study was granted by the Ethics Committee of Princess Margaret Hospital for Children.

The questionnaire included demographic information about the individual with Down syndrome and questions about the presence of current medical conditions and the extent that these conditions impacted on daily life. Information related to the use of health services in the previous 12 months, the number and reason for any hospitalisations in the previous year, and the type of illnesses experienced in the same time period was also collected. Body weight conditions were based on parental perceptions of the young person being either underweight or overweight/obese. The level of functioning in activities of daily living was measured using the Index of Social Competence (ISC).[27] With twelve subscales grouped into the domains of communication, self-care and community skills, this is an internally consistent measure of functioning which has been validated in a cohort of adults with intellectual disability.[28] Higher functioning scores indicate a higher level of functioning in daily life. The second section of the questionnaire asked mainly about family characteristics. Age was categorised into three groups: 16 to 20 years, 21 to 25 years, and 26 years and older.

### Statistical analysis

Univariate analysis of current medical conditions by age group and gender were performed. The overall and within categories of age group and gender frequency distribution of individual medical condition, and the impact of specific health conditions on daily living were explored. Pearson chi-squared test was used to test for homogeneity of proportion. Linear regression analysis was used to investigate the effect of the presence of selected medical conditions, adjusted for age and gender, on the level of communication, community and self-care skills as measured by the ISC and logistic regression to investigate relationship between some selected co-morbidities. All data analyses were conducted using Stata version 12.[29]

## Results

Of the 223 families who were invited to participate in the study, 197 (88.3%) responded. There were slightly more males (55.8%) than females in the Down syndrome sample and their median age was 23.6 years (range 16.3–31.9). Of those with living arrangements reported (n = 193), the majority (85.0%) of young adults were reported to be living with parents in the family home, 12 (6.2%) lived alone, six (3.1%) lived in a group home and six (3.1%) lived with other family or friends.

### Medical conditions

A median of four (range 0–11) current medical conditions were reported for the young adults, with slightly fewer conditions being reported for those aged between 21 and 25 years than in the other age-groups (Table 1). Eye and vision conditions were most likely to be present (in 72.6%) followed by muscle or bone conditions (in 61.1%) and body weight conditions (in 57.4%) (see Table 2).

**Table 1:** Number of current medical conditions by age group and gender.

	n	mean	sd	median	range
Overall	197	4.79	2.246	5	0–11
Age group:					
16–20 years	62	4.82	2.092	5	1–10
21–25 years	62	4.60	2.221	4	0–10
Older than 26 years	73	4.92	2.408	4	0–11
Gender:					
Male	110	4.33	2.037	4	0–10
Female	87	5.37	2.373	5	1–11

sd = standard deviation.

**Table 2:** Medical conditions overall and by age and gender of young person.

Have condition	Overall	Male	Female	16 to 20 years	21 to 25 years	26 years & over
	% (n)	% (n)	% (n)	% (n)	% (n)	% (n)
Eye/vision	72.6 (143)	69.1 (76)	77.0 (67)	69.3 (43)	80.6 (50)	66.5 (50)
Muscle/bone	61.1 (140)	74.5 (82)	66.7 (58)	77.4 (48)	71.0 (44)	65.7 (48)
Menstrual^1^	57.5 (50)	-	-	65.4 (17)	53.6 (15)	54.5 (18)
Body weight^2^	57.4 (113)	41.8 (46)	77.0 (67)	48.4 (30)	58.1 (36)	64.4 (47)
Skin	55.8 (110)	60.9 (67)	49.4 (43)	54.4 (35)	51.6 (32)	58.9 (43)
Ear/hearing	44.7 (88)	47.3 (52)	41.4 (36)	45.2 (28)	41.9 (26)	46.6 (34)
Respiratory	36.0 (71)	36.4 (40)	35.6 (31)	41.9 (26)	29.0 (18)	37.0 (27)
Mental health	31.5 (62)	32.7 (36)	29.9 (26)	33.9 (21)	27.4 (17)	32.9 (24)
Bowel	28.4 (56)	28.2 (31)	28.7 (25)	35.5 (22)	22.6 (14)	27.4 (20)
Thyroid^1^	26.4 (52)	14.5 (16)	41.4 (36)	22.6 (14)	29.0 (18)	27.4 (20)
Heart	25.4 (50)	24.4 (28)	25.3 (22)	24.2 (15)	22.6 (14)	28.8 (21)
Diabetes	1.5 (3)	2.7 (3)	0	0	0	4.1 (3)

1 only among females;

2 difference between genders p≤0.000.

Females were reported to experience more medical conditions than their male counterparts even after excluding menstrual conditions which affected more than half (57.5%) of them (Table 1). As shown in Table 2, a higher proportion of females than males were reported to have a body weight condition (77.0% vs 41.8%) and a thyroid condition (41.4% vs 14.5%). However more males were reported to have a muscle or bone (74.5%) and skin (66.7%) conditions than females (66.7% and 49.4% respectively).

There were also differences in the prevalence of medical conditions according to age. A higher proportion of the younger age group were reported to have muscle or bone conditions (77.4%), while body weight (64.4%) and skin (58.9%) conditions were more common among the older age group. In addition, menstrual conditions were more commonly reported among females in the younger age group (65.4%) and a higher proportion (80.6%) of young people aged between 21 and 25 years were reported to have an eye or vision condition than the two other age groups.

Table 3 provides a breakdown of the specific medical conditions in each category and the impact reported on the young person's daily life. More than one specific type of medical condition could be reported per category. The most common eye and vision condition was short-sightedness reported for over a third (36.5%) and considered to have an impact upon the young person's daily life in over half (55.5%). Common impacts included issues to do with safety, such as “has difficulty with daily tasks, such as negotiating steps and crossing roads” (female aged 26 years) and “can't gauge distances like crossing roads etc.” (male aged 19 years).

**Table 3:** Overall general condition and those with specific condition and the impact upon daily life.

Condition	Those with condition	Impact upon daily life^2^				
	Total	Major	Moderate	Minor	None	Missing
	% (n)^1^	% (n)	% (n)	% (n)	% (n)	% (n)
**EYE & VISION**	72.6 (143)					
Short-sightedness	36.5 (72)	8.3 (6)	22.2 (16)	25.0 (18)	16.7 (12)	27.8 (20)
Long-sightedness	23.3 (46)	6.5 (3)	21.7 (10)	34.8 (16)	19.6 (9)	17.4 (8)
Astigmatism	27.4 (54)	7.4 (4)	20.4 (11)	25.9 (14)	16.7 (9)	29.6 (16)
Strabismus	5.6 (11)	0	36.4 (4)	27.3 (3)	18.2 (2)	18.2 (2)
Other eye	17.3 (34)	8.8 (3)	11.8 (4)	26.5 (9)	11.8 (4)	41.2 (14)
**MUSCLE & BONE**	61.1 (140)					
Foot problems	63.4 (125)	5.6 (7)	24.8 (31)	35.2 (44)	12.8 (16)	21.6 (27)
Atlantoaxial instability	8.1 (16)	0	31.2 (5)	37.5 (6)	31.2 (5)	0
Scoliosis	7.1 (14)	0	7.1 (1)	64.3 (9)	21.4 (3)	7.1 (1)
Arthritis	4.6 (9)	33.3 (3)	22.2 (2)	22.2 (2)	0	22.2 (2)
Other muscle/bone	10.1 (20)	15.0 (3)	20.0 (4)	20.0 (4)	0	45.0 (9)
**MENSTRUAL PROBLEMS^3^**	57.5 (50)	10.0 (5)	32.0 (16)	30.0 (15)	0	28.0 (14)
**BODY WEIGHT**	57.4 (113)					
Obesity or overweight	57.4 (113)	9.7 (11)	29.2 (33)	27.4 (31)	8.0 (9)	25.7 (29)
Underweight	0					
**SKIN**	55.8 (110)					
Psoriasis	24.9 (49)	8.2 (4)	36.7 (18)	34.7 (17)	8.2 (4)	12.2 (6)
Acne	22.8 (45)	6.7 (3)	20.0 (9)	40.0 (18)	11.1 (5)	22.2 (10)
Fungal infections	25.4 (50)	4.0 (2)	26.0 (13)	34.0 (17)	12.0 (6)	24.0 (12)
**EAR & HEARING**	44.7 (88)					
Hearing loss	35.5 (70)	12.9 (9)	32.9 (23)	32.9 (23)	10.0 (7)	11.4 (8)
Glue ear, otitis media	15.7 (31)	6.4 (2)	29.0 (9)	35.5 (11)	12.9 (4)	16.1 (5)
Other ear	10.7 (21)	19.0 (4)	9.5 (2)	38.1 (8)	4.8 (1)	28.6 (6)
**RESPIRATORY**	36.0 (71)					
Sleep apnoea	23.9 (47)	14.9 (7)	19.1 (9)	36.2 (17)	6.4 (3)	23.4 (11)
Asthma	8.6 (17)	0	23.5 (4)	47.1 (8)	0	29.4 (5)
Other respiratory	9.6 (19)	5.3 (1)	21.0 (4)	26.3 (5)	10.5 (2)	36.8 (7)
**MENTAL HEALTH**	31.5 (62)					
Anxiety	22.3 (44)	18.2 (8)	27.3 (12)	29.5 (13)	0	25.0 (11)
Depression	11.7 (23)	21.7 (5)	21.7 (5)	30.4 (7)	0	26.1 (6)
Other mental health	10.7 (21)	38.1 (8)	9.5 (2)	9.5 (2)	0	42.9 (9)
**BOWEL**	28.4 (56)					
Constipation	23.3 (46)	8.7 (4)	37.0 (17)	43.5 (20)	0	10.9 (5)
Coeliac disease	3.0 (6)	33.3 (2)	16.7 (1)	33.3 (2)	16.7 (1)	0
Bowel other	6.1 (12)	25.0 (3)	25.0 (3)	8.3 (1)	0	41.7 (5)
**THYROID**	26.4 (52)					
Hypothyroidism	22.3 (44)	6.8 (3)	22.7 (10)	27.3 (12)	20.4 (9)	22.7 (10)
Hyperthyroidism	4.6 (9)	33.3 (3)	22.2 (2)	11.1 (1)	22.2 (2)	11.1 (1)
**HEART**	25.4 (50)					
Congenital heart disease	15.2 (30)	3.3 (1)	6.7 (2)	26.7 (8)	46.7 (14)	16.7 (5)
Cardiomyopathy	0.5 (1)	0	0	0	100 (1)	0
Other heart	10.1 (20)	0	5.0 (1)	35.0 (7)	40.0 (8)	20.0 (4)
**DIABETES**	1.5 (3)					
Type 1 diabetes	1.5 (3)	33.3 (1)	33.3 (1)	33.3 (1)	0	0
Type 2 diabetes	0					
**OTHER MAJOR CONDITIONS**	11.2 (22)					
Leukaemia	1.0 (2)	0	0	0	100 (2)	0
Epilepsy	1.0 (2)	0	50.0 (1)	0	50.0 (1)	0

1 add to more than 100% as more than one condition could be reported; ^2^not all respondents chose to answer this question; ^3^only among females.

Foot problems were the commonest muscle and bone condition reported affecting nearly two thirds (63.4%) and these were frequently (in 65.6%) reported to be impacting upon the young person's daily life. Relevant comments referred to restrictions in employment opportunities, such as “requires work that need to be seated” (male aged 20 years), and with mobility, such as “slow walker with gait affecting body aches and pains” (male aged 22 years) and “flatfooted; poor posture – walks slightly stooped and a little stiff leggedly” (male aged 19 years).

All the young adults with a body weight condition were reported as being overweight or obese and two thirds (66.4%) of parents reported that this impacted upon the young person's daily life. Common issues raised were related to mobility, such as “harder for her to get around” (female aged 27 years), “gets puffed easily” (male aged 20 years), “trouble walking distances – tires quickly” (male aged 24 years) and reduced activities, such as “participation in activity” (female aged 21 years), “not flexible, slow walker, not interested in participating in active sports” (female aged 29 years) and “lack of motivation to exercise/participate in activities etc.” (female aged 28 years). Other issues included concerns related to other medical conditions, such as “small skin lesions between thighs” (female aged 31 years) and “obesity caused his knee caps to dislocate, limping most of the time especially in winter” (male aged 28 years).

One half (55.8%) of parents reported that the young adult had a skin condition with 25.4% reporting fungal infections, 24.8% psoriasis and 22.8% acne (see Table 3). A slightly higher proportion (79.6%) of parents reported that psoriasis impacted on their young person's daily life compared with acne and fungal infections (65.9% and 64.0% respectively). Embarrassment issues were also raised for those with psoriasis, such as “wears long sleeves and pants due to embarrassment” (female aged 30 years).

While just over half (57.5%) of the young women were reported to have a menstrual condition, almost three quarters (72.0%) of parents reported that these conditions impacted on the young woman's life. Comments included issues related to attending employment, such as “has to have days off work” (female aged 25 years) and “sometimes not able to attend work” (female aged 19 years), to hygiene, such as “does not manage periods well – doesn't change pads often enough” (female aged 26 years), and to activities, such as “has low pain threshold sometimes misses activities” (female aged 19 years).

Although less than one third (31.0%) of the young people were reported as having a mental health condition, a large proportion (74.4% for anxiety and 73.9% for depression) of parents reported that this impacted upon the young person's daily life (Table 3). Comments from parents among young adults with anxiety include “extreme anxiety effects every aspect of life: work, leisure, friendships” (female aged 25 years), “anxious about future, often refusing to do things” (male aged 17 years), “worries a lot, gets headaches and does not sleep well” female aged 27 years), “dwells on things unnecessarily” (male aged 22 years), and “doesn't want to go out in public” (male aged 25 years). Among those reported to have depression comments included “unable to function without medication” (female aged 29 years) and “work hours reduced. Social activities reduced. General wellbeing flat” (male aged 24 years).

While one quarter (26.4%) of young people were reported to have hypothyroidism, young adults who were reported as being overweight or obese were 2.9 times more likely (OR 2.88; 95% CI 1.42–5.84) to have a thyroid condition than those who were not overweight or obese. Furthermore, females were four times more likely to have a reported thyroid condition (OR 4.15; 95% CI 2.10–8.19) than males. Over half (56.8%) of parents with young people with hypothyroidism reported that there was an impact upon the young person's daily life. Comments reported by parents included issues related to lethargy, such as “without taking the medication he would be too lazy to move around” (male aged 28 years). One parent reported a number of issues which highlights the complexity of providing care to this population “As he has a phobia of hospitals and needles, the only way we can get blood to test his levels is when he has an anaesthetic. He has not had blood levels done for 5 years as we are unable to restrain him despite large doses of lorazapam. His skin and hair are extremely dry. Constipation a problem. Falls asleep frequently during the day, but consultant reluctant to increase thyroxine further without blood levels.” (male aged 25 years).

### Level of functioning and health conditions

The young adult's level of functioning was measured using the ISC [28] and included three skills domains of communication (mean 5.66, sd 1.52, median 6, range 2–8), community (mean 11.05, sd 4.28, median 11, range 4–19) and self-care (mean 19.92, sd 4.18, median 20, range 7–26). After adjusting for gender and age, young adults with mental health conditions were more likely to score lower on communication skills (−0.57, 95% CI −1.02, −0.13), community skills (−1.36, 95% CI −2.63, −0.09) and self-care skills (−1.99, 95% CI −3.21, −0.78) than those without a mental health condition (Table 4). There were no other strong relationships found between the remaining health conditions and level of functioning scores.

**Table 4:** Linear regression analysis of specific medical condition and level of functioning^1^.

	Measures of functioning^2^					
	Communication skills		Community skills		Self-care skills	
Have condition	Coef.	95% CI	Coef.	95% CI	Coef.	95% CI
Mental health	−0.57	−1.02, −0.13	−1.36	−2.63, −0.09	−1.99	−3.21, −0.78
Respiratory	−0.49	−0.92, −0.05	−0.83	−2.06,0.40	−1.26	−2.45, −0.06
Ear/hearing	−0.49	−0.91, −0.08	−0.22	−1.41,0.98	−0.71	−1.87,0.45
Skin	−0.32	−0.74,0.10	−0.20	−1.39,0.99	−1.16	−2.31, −0.01
Bowel	−0.44	−0.90,0.03	−0.42	−1.74,0.90	−1.39	−2.66, −0.12

Coef.  =  Coefficient.

1 Adjusted for gender and age; ^2^Coefficients are not comparable between different domains of functioning due to the different scales of each domain.

### Recent illness, hospitalisations and health care provider visits

The most common acute illnesses reported in the previous 12 months were cold or influenza (experienced by 74.0%, median episodes 2, range 1–20) and ear infection (experienced by 22.7%, median 2, range 1–12). Thirty seven of the young adults (20.7%) had at least one hospital admission (median admission 2, range 1–3) and common reasons were for surgery (n = 8), dental treatment (n = 8) and eye treatment (n = 7).

A total of 174 (88.3%) young people had visited their general practitioner in the previous 12 months (median number of visits 3, range 1–15), 20 (10.1%) visited a psychologist (median 5, range 1–20) and 14 (7.1%) a mental health doctor (median 2, range 1–12). Information was also provided about other specialist services used by the young adults in the previous 12 months. A total of 92 (46.7%) had visited “other specialists” that included: 25 (12.7%) visiting an eye specialist, 24 (12.2%) an ear nose and throat specialist and 21 (10.7%) a dentist. A range of allied health professionals were also visited by 45 (22.8%) of whom 13 (6.6%) visited a podiatrist. Eighteen (9.1%) were reported having visited “alternative therapists” of which five visited a naturopath.

## Discussion

This is the first paper to our knowledge to describe both the prevalence of medical conditions and their impact in a population of adolescents and young adults with Down syndrome. We previously examined the prevalence of medical conditions in school-aged children with Down syndrome in 1997[23] and 2004[22]. In 1997 we found that eye or visual problems were the commonest condition experienced by 75% with current problems in 43%, followed by ear or hearing problems experienced by 57% and with current problems in 23%. Cardiac problems had affected 40% but only 7% had current problems and bowel problems 21% with current problems also in 7%. Finally, thyroid disease was reported for 14% with current problems in only 6%. When we compared the 2004 with the 1997 data we found that in 2004, children with Down syndrome were less likely to have a current problem due to their cardiac condition but more likely to have a bowel condition reported but that there was an overall reduction in episodic illnesses and infections. If we compare the prevalence of health conditions in adolescents and young adults (from the current study) with that of school-aged children at the previous time point (2004)[22], as illustrated in Figure 1, the main differences we see are in the increased prevalence of musculoskeletal problems in young adults 61% compared with only 36% in the school-aged group and of thyroid problems 26% vs 13%. In contrast the main decreased prevalences we see are in respiratory conditions reported in 60% of the school-aged group but only in 36% of the young adults and in heart conditions from 46% in the school-aged to 25% in the young adults. In the school-aged surveys just over a third (39%) of families commented on difficulties in experiencing a healthy weight (unpublished data) compared with 57% of the young adults in the current study. We did not previously specifically ask questions about mental health but the figure of a prevalence of nearly a third in the current study is concerning. We also noted a decrease in episodes of acute illness. Only 74% were reported to have an episode of influenza compared with 85% in the 2004 school-aged cohort (unpublished data), 23% an ear infection compared with 30% and 21% a hospital admission compared with 31%.

**Figure 1:** Prevalence of specific medical conditions in children with Down syndrome at school-age and young adults. Black dot: Cardiac. Black diamond: Bowel. Vertical line: Ear/hearing. Black square: Eye/vision. X: Thyroid. Upside-down black triangle: Musculoskeletal. Black triangle: Respiratory.

Aside from the survey data obtained from our population cohort we have also previously studied the morbidity patterns in children with Down syndrome through hospitalisation linked data.[30], [31] Here we found that upper respiratory tract conditions affected the most children (58%) and accounted for 12% of all admissions. Other disorders, which affected a high percentage of children, were ear/hearing conditions (51%), lower respiratory tract conditions (37%) and disorders of the oral cavity (38%). Overall, we were able to demonstrate that children with Down syndrome were being hospitalised at a rate five times that of the general population. Therefore the health profile of the adolescents and young adults presented through this current study would appear to be somewhat different from that of their younger peers in that they probably have fewer acute episodes of illness, especially respiratory infections and less need for hospitalisations. However in contrast, they would appear to be developing more life style diseases such as obesity, mental health and musculoskeletal problems.

The high prevalence of overweight and obesity which we identified and has previously been reported[32] is of concern. In particular the impact of being overweight on motivation and ability to participate in physical activity, which would help prevent and manage weight gain, is worrisome. Overweight and obesity are linked with an increased risk of type 2 diabetes, commoner in Down syndrome[33] although not identified in our cohort, as well as cardiovascular disease and cancer. Obesity can also exacerbate some gastrointestinal and orthopaedic conditions, impacting further on quality of life among this group.[34] An association has been reported between a reduced body-mass index and lifestyle variables including satisfaction in friendships and access to social and recreational opportunities for adults with Down syndrome.[35] Recent research has emphasised that support workers can play a key role in encouraging participation in physical activity for this group.[36], [37] It has also been suggested that, similar to many people without impairment, adults with Down syndrome often lack the motivation to exercise as well as being restricted due to medical and physiological factors. Research into factors impacting on the body composition of young people with Down syndrome is currently underway by our study team.

Consistent with previous research raising concerns about the mental health of people with intellectual disability,[38], [39] we found mental health conditions to be almost four times higher than in the general WA population of similar age.[40] The prevalence of depression in our cohort was similar to that reported in previous studies of people with Down syndrome (16% for depression and/or anxiety;[41] 11% for one or more episodes of depressive illness;[42] and 22% for emotional problems[32]) but higher than reported among adults with Down syndrome based on clinical diagnostic criteria (3%).[43] In our study mental health conditions were reported to have an adverse impact on employment as well as leisure and social activities among the young adults. We also found that those with mental health problems scored lower on all three measures of functioning, although the directionality of this association is not able to be determined due to the cross-sectional study design. That is, we do not know whether mental health conditions impacted levels of functioning or whether level of functioning impacted on mental health conditions. Further research is needed to determine the prevalence, predictors and impact of mental health conditions in people with Down syndrome.

Muscle and bone conditions had double the prevalence in this young adult cohort compared with our findings in childhood and can be exacerbated further by obesity and inactivity.[22] Foot problems were the most common condition and their frequency appeared to be increasing. These conditions were reported to have an impact on both employment and mobility and yet only 7% of the total sample had been reported to visit a podiatrist in the previous year.

The prevalence of skin conditions in our cohort was much higher than reported previously among young people with Down syndrome aged between 0 and 29 years.[41] More than two thirds of our parents reported that these conditions impacted on the young person's daily life and those with skin conditions scored lower on self-care skills. There is a need for more research into both the treatment of skin conditions and the impact upon daily life.

There has been minimal research [44] into the prevalence and impact of menstrual conditions among young women with Down syndrome. Nevertheless, menstrual issues have important impacts upon daily activities including restrictions on employment and social participation, as well as issues related to hygiene needs among these young women. Furthermore, previous research among parents and carers of women with intellectual disability found that menstrual problems were no more common in this group than in the general population, but may be experienced more negatively and not always appropriately recognised.[45] Further research is needed to develop optimal strategies for menstrual management for young women with Down syndrome and other intellectual disability.

We have shown in our population-based Down syndrome cohort that the prevalence of thyroid disease increases with age at least into early adulthood. The prevalence of hypothyroidism among children with Down syndrome has been reported to range between 8% and 28%. [41], [46], [47] We also found gender differences with young women four times more likely to be reported to have a thyroid condition and those who were reported to be overweight and/or obese almost three times more likely. That there were impacts reported by parents for just over half of the young adults raises the question as to whether this condition is being adequately monitored and maintained for this group. These findings support the need for young people to have their thyroid levels regularly checked and treatment initiated and monitored if a thyroid condition is detected.

Overall there is limited research on the extent of health service use by other populations of young people with Down syndrome with which to compare our findings. However, In a US study using hospital records there was an average of two (range 1–3) health care sub-specialities being accessed by adults with Down syndrome transitioning from child to adult care.[48] When compared to the general Western Australian population aged between 15 and 24 years,[49] hospitalisations were higher in our Down syndrome cohort (21% versus 9%) while general practitioner visits were similar (72% versus 76%) and dentist visits were lower (11% versus 47%). In contrast, other sources report that between 50%[41] and 68%[50] of young adults with Down syndrome had visited a dentist in the previous year. However, dentists were not included as a separate medical specialist in the questionnaire and thus their visits may have been under-reported in our results.

While many of the conditions we identified among young adults with Down syndrome are also seen in the general population, these young people experience multiple conditions and, often, at a higher prevalence. Eye and vision, muscle and bone conditions, menstrual conditions among young women, body weight, skin, ear and hearing, respiratory and mental health conditions were each reported to affect one third or more of our cohort. Furthermore, some level of impact upon the young person's daily life was reported with few parents reporting no impact across these conditions. These parent-reported impacts included restrictions in opportunities to participate in employment and community leisure activities for the young people, as well as safety concerns although we did not demonstrate any impact of medical conditions on participation when we previously described friendships and leisure activities in children with Down syndrome.[51]

To our knowledge, this is the first study to report the comprehensive list of medical conditions experienced by young people with Down syndrome and the impact upon their daily lives. Furthermore, it is among the first to report on the use of medical and health services by this group. There has been no validation of the reported conditions with medical examinations or clinical measures and body weight conditions reported by parents were not validated with biometric measures. However from the health assessment literature it is clear that the identified health needs, be it morbidity or unmet health screening/promotion, exist and the level of comorbidity reported by the parents underestimate the real prevalence of disease experienced by this population.[52], [53]

An additional strength of this study is the inclusion of a large representative cohort of community-living young Western Australians with Down syndrome with a good response fraction. However there are some limitations that require noting. While the questionnaire collected comprehensive information related to many aspects of the young person's life, it was long and could have resulted in respondent fatigue. There may also have been a level of recall error associated with retrospective parent-report although it was mostly related to fairly recent events. These two aspects may have contributed to missing data that limited the interpretation of some of the findings. Of note were the data missing in relation to the level of impact of medical conditions and, among those who did report, often there was no indication of how this was impacting. However, parents were encouraged to complete the questionnaire in their own time and at multiple sittings. They were also provided with options to complete a web-based or paper version of the questionnaire or by telephone or face-to-face with a research team member.

The cross-sectional nature of the study limits conclusions and directionality. As such, there is no indication of the influence of the functional scores upon the health conditions or whether the health conditions influenced the functional scores.

## Conclusion

Monitoring and screening for health conditions among young adults with Down syndrome is important due to the number of conditions that occur among this group. This will assist with developing management plans and strategies to avoid long-term consequences of these conditions and to ensure that they do not act as barriers to participation in employment and social activities. There is also the need to develop and implement strategies and programs that promote healthy lifestyles among young people with Down syndrome.
